The article "Research on Athlete Detection Method Based on Visual Image and Artificial Intelligence System" was retracted in 2023. Reasons: signs of a paper mill; suspected computer-generated content; unreliable results or conclusions; concerns about the data.

# Research on Athlete Detection Method Based on Visual Image and Artificial Intelligence System

**DOI:** 10.1155/2022/2418367

**Published:** 2022-09-29

**Authors:** Weiyi Wang

**Affiliations:** Baotou Medical College, Baotou, Neimenggu, China

## Abstract

Pedestrian detection and tracking based on computer vision has gradually become an international pattern recognition, which is one of the most active research topics in the field of computer vision and artificial intelligence. Using the theoretical results in the field of pattern recognition and computer vision technology, we are committed to detect and track pedestrians from video sequences. In addition to computer vision-based passer-by detection and tracking technology as the key, in the advanced computer vision action and analysis, it has a direct impact on the accuracy and robustness of its understanding. We analyzed various targets, such as subsequent recognition motion and pedestrian motion, and described them as high-level application processing, such as action understanding. In addition, because of the unique texture of human clothes compared with the surrounding natural landscape, they are highly “prominent” from the perspective of human visual system, and they are particularly prominent in the peripheral part of human contact with the background. In this paper, a binary function based on importance is proposed. As the space representation of image itself is not sensitive to noise and local signal, space representation is used. In addition, as an observation model, it can reduce the adverse effects of background noise and local noise on the tracking algorithm. Through the function block tracking, the pedestrian's body can be tracked in detail. At the same time, the color band learning method is used to update the target template online to deal with the changes of target appearance caused by sunshine, pedestrian posture, and other factors. According to the experimental results, even if the appearance and posture of pedestrians change greatly, it has a stable tracking effect.

## 1. Introduction

Humans perceive the world mainly through eyes and ears, and the brain further analyzes, understands, and judges the sensed information. Studies have shown that when humans perceive and understand the surrounding environment, more than 80% of the information comes from the visual system [1]. It is said that “a picture is worth a thousand words.” Among the various pieces of information that humans perceive from the outside world, visual information is not only intuitive and easy to understand but also contains a lot of information [2]. Therefore, in many cases, a single image is more informative than a word. Nowadays, as mankind enters the computer age, computers cover almost all areas of human production and life, affecting and changing people's lifestyles [3, 4]. To enable computers to provide better services to humans and to interact smoothly with humans, the visual function of computers is to recognize and understand the world through the same visual system as humans and be able to independently judge and create the environment [5].

## 2. Related Work

In the past ten years, literature on pedestrian detection and tracking based on computer vision has become one of the most active international research topics in the field of pattern recognition, computer vision, and artificial intelligence [6]. The core of the literature is to combine computer vision technology and use theoretical results in the field of pattern recognition to detect and track pedestrians in video sequences [7]. Literature is the basis of computer vision's more advanced behavior understanding analysis [8]. Its accuracy and robustness are used in various advanced application processing, such as target recognition, pedestrian motion analysis, behavior description, understanding, etc. Therefore, pedestrian detection and tracking based on computer vision are more like intelligent video surveillance, intelligent transportation, car driving assistance, advanced human-computer interaction, action-oriented behavior analysis, virtual reality, and so on [9]. It is the foundation of advanced applications. Literature can obtain information, such as the position, speed, direction, proportion, and posture of pedestrians, by detecting and tracking pedestrians, and upon comprehensively analyzing and processing this information, more advanced pedestrians can be obtained [10]. One can get a description and understanding of the action. The intelligent video surveillance system mainly sends the video sequence captured by the imaging device to the computer. The document determines the system when analyzing and judging the video sequence according to predetermined rules, and if there is normality that violates the rule, phenomena like the long-term stay of pedestrians occur [11]. The system will automatically send alarms so that security personnel can respond to these abnormal situations quickly and effectively. Virtual reality is an integrated technology that integrates many fields by detecting and analyzing the human body in the image [12]. Literature realizes the three-dimensional model of the human body by combining other information and performing a large number of calculations, and it synthesizes the three-dimensional image of the human body, which is a new way for computers to interact with people [13]. In the past ten years or so, the field of pedestrian testing has achieved rapid development in various methods and technologies, has made considerable progress, and achieved better test results under certain restrictions. Some technologies have been successfully applied in the real world. The literature must clearly recognize that the general human body detection has a variety of postures, the color and texture of the clothes are widely scattered inside, the background caused by camera movement changes, there is mutual shielding among pedestrians in crowded environments [14], etc. Detection has received extensive attention in the field of computer vision. For example, some papers at the 2013 international conference CVPR were still studying pedestrian detection.

## 3. Analysis of Athlete Detection Algorithm Based on the Visual Image

### 3.1. Detection Algorithm Based on RANCS and SBF Features and Fern Classifier

Naive Bayes classifier is a supervised learning method that assumes the influence of attribute values on a particular class and makes it independent of other attribute values. However, this restriction is very strong and usually unsatisfactory. Later, Ozi Sal et al. put forward the concept of “half-Neibes embrittlement,” which is also called “random fern classifier” in the literature. Conceptually, the Landafern classifier is a variant of the Landafern classifier that has been very successful in the fields of visual object tracking, object recognition, and image classification in recent years. It has the characteristics of high accuracy, high efficiency, low classification error rate, and high classification speed. For example, Kalal et al. used the Randfern classifier in the document to reliably track the target in real time, while ozuysal et al. used the Randfern classifier in the document [10] to quickly identify important points and achieve high-precision key matching. The following will further describe the principle of the random hair classifier to easily understand the life classifier. The following is based on the detection of passers-by, and the law is set to zero, i.e., as a nonhuman body or a human body, it extracts samples of candidates and waits in the same way. After the maximum value of the candidate samples that can be obtained in the category, the test probability is classified.

(1) $$\begin{array}{c} {\hat{c}}_{i}=\underset{c_{i}}{\text{argmax}}P\left(C=c_{i}\left|f_{1},f_{2},\ldots ,f_{N}\right.\right). \end{array}$$

Among them, *C* refers to the category, according to the Bayesian rule.

(2) $$\begin{array}{c} P\left(C=c_{i}\left|f_{1},f_{2},\ldots ,f_{N}\right.\right)=\frac{P\left(f_{1},f_{2},\ldots ,f_{N}\left|C=c_{i}\right.\right)P\left(C=c_{i}\right)}{P\left(f_{1},f_{2},\ldots ,f_{N}\right)}\\ {\hat{c}}_{i}=\underset{c_{i}}{\text{argmax}}P\left(f_{1},f_{2},\ldots ,f_{N}\left|C=c_{i}\right.\right)P\left(c_{i}\right)\text{.} \end{array}$$

For pedestrians and non-pedestrians, the prior probability follows the average distribution. Hence, the formula can be simplified.

(3) $$\begin{array}{c} c_{i}=\underset{c_{i}}{\text{argmax}}P\left(f_{1},f_{2},\ldots ,f_{N}\left|C=c_{i}\right.\right)\\ P\left(f_{1},f_{2},\ldots ,f_{N}\left|C=c_{i}\right.\right)=\overset{N}{\underset{j=1}{\Pi }}P\left(f_{j}\left|C=c_{i}\right.\right)\text{.} \end{array}$$

Usually, this assumption is wrong. Upon considering the relationship between the features, the comparison of the inadequate equation and the probability after the test will provide a compromise solution for the proper solution of the hesitation problem. According to each sample test, the features of n are divided into m groups, the features of m are included in each group, and the single life classifier corresponding to each group, the total m life classifier is all conditions. Calculate the probability of the *m* team.

(4) $$\begin{array}{c} P\left(f_{1},f_{2},\ldots ,f_{N}\left|C=c_{i}\right.\right)=\overset{N}{\underset{k=1}{\Pi }}P\left(F_{k}\left|C=c_{i}\right.\right)\text{.} \end{array}$$

Among them, *k* represents the characteristic random sequence function of the *k* team, which is a combination of the characteristics of the function. In this process, the characteristics of each group will be randomly distributed. Regarding the characteristics of the last 1 *k* team, the similar conditional probability of the corresponding life classifier is kf)) kipfc=c.

(5) $$\begin{array}{c} p_{k_{f_{i}}}=\overset{N}{\underset{k=1}{\Pi }}P\left(F_{k}\left|C=c_{i}\right.\right)=\frac{N_{k_{f_{i}}}^{l}}{N_{c_{i}}}\text{.} \end{array}$$

Among them, the number of training samples of type *i* is the classification of samples of *k*. The feature of the team corresponds to the number of training samples of the leaf node of life classifier 1, and the value of *l* is the second-level feature corresponding to the fruit of the classifier. For each node and each life classifier, the number of samples of the node is similar to the number of training samples. This value can be 0 because there are not enough training samples during training. Therefore, replace the above formula with the following formula:

(6) $$\begin{array}{c} p_{k_{f_{i}}}=\frac{N_{k_{f_{i}}}^{l}+N_{r}}{N_{c_{i}}}\text{.} \end{array}$$

Usually, the value of this decree is 1. After extracting features from the sample to be detected in combination with pedestrian detection, *r*_*n*_ can obtain the classification result by the following formula:

(7) $$\begin{array}{c} {\hat{c}}_{i}=\underset{c_{i}}{\text{argmax}}P\left(f_{1},f_{2},\ldots ,f_{N}\left|C=c_{i}\right.\right)=\underset{c_{i}}{\text{argmax}}\left(\overset{M}{\underset{k=1}{\Pi }}P\left(F_{k}\left|C=c_{i}\right.\right)\right)\text{.} \end{array}$$

The author has briefly introduced the fern classifier. To understand its classification principle, the author will introduce a specific example (the author will further introduce the above example. Below, some images are used to illustrate sample features. Specific examples, such as extraction and describing training methods, are used to describe single fern classification, the classification method, and the single fern classifier.

#### 3.1.1. Binary Feature Extraction

(8) $$\begin{array}{c} \frac{f_{1}=I\left(x_{a},y_{a}\right)>I\left(x_{b},y_{b}\right)⟶true⟶1}{f_{2}=I\left(x_{c},y_{c}\right)>I\left(x_{d},y_{d}\right)⟶false⟶1}\text{.} \end{array}$$

According to the rules of the formula above, it can be represented by the mapping between binary and decimal numbers, as shown in Figure 1.

#### 3.1.2. Training a Fern Classifier

The above picture is another form; the number in the book is 5, and training is a separate existence. The graph of the classifier, firstly, sorts the samples of each training and randomly classifies the intermediate values. The mapping of each sample obtained by the rule of the equation is the following figure. Pay special attention to the binary value here. When random, after fixing the sample position, all training and testing sample positions will be modified in the future. Secondly, the decimal mapping obtained by each training sample corresponds to various mappings based on the decimal value of each training sample, and finally, the number of training samples is calculated. Statistically, please refer to the following formula for the value of bin.

#### 3.1.3. Multiclass Single Classifier

As shown in Figure 2, the training number is from 0 to 9 of the digital sample photos. There are 5 training samples, divided into 10 types in total. For each numerical sample class, train each fern classifier in the same way as in (2), and there are 10 training results on the right. This figure shows the classification process or classification process after the largest sample is found by the fern classifier when a single test sample is given.

Firstly, extract the binary features from the test sample, and find the corresponding decimal value. Then, get the value of the corresponding bin among these 10 types from each decimal value. Finally, the formula in the figure below gives the largest trailing class.

(9) $$\begin{array}{c} {\hat{c}}_{i}=\underset{c_{i}}{\text{argmax}}P\left(C_{i}\left|F\right.\right)=\underset{c_{i}}{\text{argmax}}\left(F\left|c_{i}\right.\right)\cdot P\left(C_{i}\right)\text{.} \end{array}$$

In the formula, various prior probabilities are the same under normal circumstances. Above, we introduced an example of a multiclass single classifier; however, in Section 3.1.4, we will introduce a fern classifier using semisimple Bayes.

#### 3.1.4. Semisimple Bayesian Classifier

When applied in practice, it turns out that a single fern classifier is not enough for classification, and the concept of random multiple far classifiers has been proposed. At that time, a total of 5 *n* 15 binary features were extracted from the numerical training samples, and these 15 features were divided into *m* 3 random sets. Each feature group corresponds to one fern classifier, and there are 3 fern classifiers in total. Finally, a random fern classifier can be used to obtain the largest postclassification.

(10) $$\begin{array}{c} {\hat{c}}_{i}=\underset{c_{i}}{\text{argmax}}\left(\overset{M}{\underset{k=1}{\Pi }}P\left(F_{k}\left|C=c_{i}\right.\right)\right)\text{.} \end{array}$$

In short, compared with a single fern classifier, the semisimple bay-based random multifur classifier actually divides each sample feature into multiple groups. These groups correspond to a single category of ferns. After division, the posterior probability of the sample is equal to the product of the posterior probability of a single Fern classification.

Image importance detection is an important field of computer vision research. Its basic idea is to simulate the attention and analysis process of scenes seen by human vision and arouse further attention to visual scenes. These areas of interest are captured through the bottom-up and top-down models. For the bottom-up model, the salient features of certain image areas are excellent, which are mainly attributed to the features at the bottom of the image itself, such as strong color adjustment and contrast in the image and unique shapes compared to the surrounding environment. The obvious sex zone is an element of personal taste and emotion. The image will not be mixed with people, thus forming a competitive contrast between its bottom features. In the bottom-up model, the acquisition of important image areas is directly related to the observer's prior knowledge and the observer's purpose and interest. For example, different people may obtain different attention results in the same scene for the same purpose.

In the bottom-up visual attention calculation model, because of the salient nature of the image, the normal generation can cover an important gender area map. In the two-dimensional “image” with the same correspondence relationship with the image, the value of each pixel is the saliency of the original image, and the intermediate value is larger. “The greater the saliency of the same area in the original image, the more the number of humans. Gathering visual attention: the importance map contains two types of information. It can provide the scale information of important areas and the spatial distribution of importance in the image, as shown in the figure.  Figure 3(a) is the original input image, 3(c) is the importance map, 3(d) is the heat map formed by the intensity of importance in the importance map, and red is more important. As shown in the figure, it is the saliency area extracted with a certain limit value according to the saliency map. As shown in the figure, the saliency area detected by the computer vision technology is human. It almost coincides with the area considered important by vision.

With the continuous in-depth research of computer vision technology, related mature technologies are increasingly used in real-world production and life, and the visual selective attention mechanism is increasingly attracting widespread attention from researchers in the field of computer vision. The extraction of effective image area is widely used in image retrieval, image classification, and object recognition. The pedestrian feature extraction algorithm based on importance will be described in detail below. To detect passers-by, the characteristics of human clothing, the surrounding relatively natural colors, the unique color characteristics and texture characteristics of the scene, it is caused by the outline of the human body and the unique left-right symmetry and upright characteristics. Because of these characteristics, the surrounding natural scenes are also “important.” Hence, the bottom-up model is suitable for detecting contour edges when leaving people. In the process of extracting human features based on saliency introduced in this section, the saliency detection algorithm is mainly used to extract human contour features, and then the human feature descriptors are extracted from the contour features. In the following, we will introduce a method for human body binarization feature extraction based on importance detection algorithm.

It is a simple calculation model of the visual importance of an image. The core point of this article is that from the point of view of information theory, information is divided into redundant parts and changing parts. Human vision is very sensitive to changing parts. One of the basic principles of the visual system is to be sensitive to nontraditional features while suppressing responses to frequently appearing features. Therefore, the image can be divided into the following two parts:

(11) $$\begin{array}{c} H\left(\text{im}age\right)=H\left(innovation\right)+H\left(prior\;knowledge\right)\text{.} \end{array}$$

We also propose that the average of the logarithmic spectrum of a large number of images is proportional to the reciprocal of the frequency obtained by taking the natural logarithm of the amplitude spectrum after the Fourier transform of the image.

(12) $$\begin{array}{c} E\left\{A\left(f\right)\right\}\propto \frac{1}{f}\text{,}\\ R\left(f\right)=L\left(f\right)-A\left(f\right)\text{,}\\ A\left(f\right)=R\left(F\left[I\left(x\right)\right]\right)\text{,}\\ P\left(f\right)=R\left(F\left[I\left(x\right)\right]\right)\text{,}\\ L\left(f\right)=\log\left(A\left(f\right)\right)\text{,}\\ R\left(f\right)=L\left(f\right)-h_{n}\left(f\right)*L\left(f\right)\text{,}\\ S\left(x\right)=g\left(x\right)*F^{-1}{\left[\exp\;\left(R\left(f\right)+P\left(f\right)\right)\right]}^{2}\text{.} \end{array}$$

In addition to the unique bilateral symmetry and uprightness of human beings, compared with the surrounding natural landscape, human clothes also have a unique texture and color. These characteristics are strongly “prominent” for the author and the natural landscape. In addition, the part where the human body is in contact with the background, i.e., the edge and background of the human body, is an area that is “important” to the human visual system and can be visually attracted. The significant detection method is used to obtain the contour of the human body on the human test sample. As shown in the figure, (a) is the original image, (b) is the effective image, and (c) is the corresponding heat image. The outline of the human body can be clearly identified from the image, i.e., important detection is very effective for detecting the contour of the human body in the sample image of the pedestrian.

In order to illustrate the effectiveness of the effective detection of the extracted human contour and display the statistical features, that is, the extracted contour well represents the contour features of the pedestrian, as shown in the figure, the contour map is accumulated and the statistical features similar to the histogram features in the gradient direction of the average value are created. Using the MIT pedestrian database as a test sample, an effective detection algorithm based on spectral residuals is used to perform effective detection, and an effective map including the contour of the human body is obtained.

The figure shows the effective detection of positive test samples based on the effective detection algorithm based on the spectral residuals and obtains the average effective map including the contour of the human body, which is positive in the pedestrian database of the Massachusetts Institute of Technology. The effective images of 10 frames, 20 frames, 30 frames, 50 frames, 100 frames, and 300 frames before the sample average are listed, respectively. It can be seen from the figure that although the average saliency gender map contains only 10 samples, the contours of the body are depicted very well, and the average saliency gender map also contains 50 samples. And it contains 100 samples. The significant gender maps of 300 samples are basically the same. In other words, the significant gender profile of the samples detected in the human body is good and has strong characteristics, scattered in less uniform categories, and it effectively outlines the upright characteristics and bisymmetric and horizontal differentiation. It is the average value of the gradient plot, containing positive samples from humans. In this paper, the gradient of a given positive sample is first dalsketch, and then the average of these gradient graphs. In the same way, in the MIT passer-by database, the sample before the sample 10 frames, 20 frames, 30 frames, 50 frames, 100 frames, and 300 frames, the average gradient acquisition results are shown in the figure. It can be seen from the figure that even if the outline of the human body is drawn, the average gradient map is good, however, because of statistical characteristics, our needs are much more obvious than the average gender map, contours, and backgrounds with average gradient people. The contrast between the outline of the average extraordinary person we introduced and the background is slightly different, i.e., the outline is obvious. The reason for this phenomenon is that the outline of the human body is prominent, and the outline of the display content is emphasized as a feature. The feature of the details is that it is the entire gradation map, and the feature of the human body contour is not “important.” As a result of pedestrian inspection, even if it must have attributes that can reflect the essence of the human body, it is characterized by strong linearization, i.e., strong partitioning, and it is a feature that satisfies the contours of the human body. Because of this characteristic, the slope in the figure does not have detailed features, such as cracks on the clothes, which are relatively different for pedestrians in the texture of various clothes, the dispersion within the category, and the larger extraction. For contour features, the contours of the human body based on the significant gender are more obvious, and the characteristics of the human contours are more prominent.

Figure 3 shows the significant detection of positive test samples based on the saliency detection algorithm based on spectral residuals, and the average saliency map, including the silhouette of the human body is obtained, as shown in the figure. The average value of important blueprints such as trees, buildings, lakes and forests is important. The average of 10 frames, 50 frames, 100 frames, and 300 frames randomly sampled by pedestrians in the database is listed in the significant blueprints. It can be seen from the figure that even an average saliency map containing only 10 positive samples can well-depict the outline of a person. We recommend extracting the outline of a person based on the saliency. Features can describe a person's silhouette very well. It can be seen from the figure that natural landscapes do not have the uniform characteristics of human silhouettes. Hence, their average prominence maps are chaotic and have no statistical rules. It shows that the human profile feature distinguishes the background from other purposes better than other features.

In the following, we introduce the basis of the saliency chart and extract the binary features, as shown in the figure. Firstly, obtain the marked chart in the figure through the saliency test, and then proceed to the saliency Laguna Beach. In this figure, when it is random, the new intermediate adjustment value of the red time at any time is n()rixy, where the intermediate adjustment value is the subpixel of the 7 × 7 size image centered on the red dot. The intermediate adjustment value of the blue time is isbixy, and similarly, the intermediate adjustment value here is the intermediate adjustment value of the subelement of the 7 × 7 size image centered on the blue dot. For any point, the conditions to be satisfied are as follows:

(13) $$\begin{array}{c} \frac{f_{1}=I_{r}\left(x,y\right)\geq I_{b}\left(x,y\right)⟶ture⟶1}{f_{2}=I_{r}\left(x,y\right)<I_{b}\left(x,y\right)⟶false⟶0}\text{.} \end{array}$$

The point to be emphasized here is that the position of the graph is in the figure. Firstly, set the generation time position according to the generation of the part of the standard with good random algorithm. However, in the subsequent training, the positions of these points are fixed in all subsequent samples and test sample extraction feature vectors, and the order of forming the binary vector category at one time is also preset.

### 3.2. Experimental Results and Analysis

In the experimental analysis stage, the dataset of the French National Institute of Information Automation and the dataset of the Massachusetts Institute of Technology are used as the database for pedestrian training and testing. Moreover, the samples that match the pedestrian scale of MIT will first collect and test the database training samples and then reduce the size of the positive samples to 128 × 64. In order to train, collect, and test two databases, sample images with random resolution are lost. In these two databases, many scenes with missing sample images are usually natural, roads, buildings, and other backgrounds.

When selecting pedestrian characteristics, compared with natural scenes, there are overall consistent characteristics in clothing based on the appearance or shape of pedestrians and the two geometric symmetries. Compared with other target categories, it adds unique pedestrian characteristics, such as a unique texture and a unique silhouette, when a pedestrian stands upright. Using the introduced random color similarity function (rancs) and the introduced importance-based binarization function (sbf), the classification method is explained. Use the introduced Landfern classifier to train and classify training samples and test samples. Before training the classifier, the random color similarity (random number) function has a lot of work to do. The parameter adjustment experiment must be repeated, such as pixel size and position. These optimization experiments are very important, and the successful combination of parameters can greatly improve the effectiveness of feature classification. In order to obtain the best parameter Union, the pixel sizes 4x4/7x7/10x10/12x12/13x13 are tested. In some cases, select the level when constructing the histogram, such as 8/10/12/16; each color segment is tested, and the minimum distance between the selected cells is 3/5/ 7. If so, get the final highest parameter set. As for the parameter combination used in the experiment, the number of stages of the histogram of the rgb color space is 16 × 16 × 16, the pixel size is 7 × 7, and the minimum distance between the pixel pairs is 7 pixels. For importance-based binary functions (sbf), the importance algorithm is an importance detection algorithm based on spectral residuals, and the gray value of a random point is that the center of the point is 7 × 7. Using the average gray value of image sub-blocks, the shortest distance between each pair is 7 pixels.

Color similarity (rancs) features are randomly selected, and the extracted feature size of each sample is 500, i.e., the position of the sample image is preselected according to the image unit, and 500 pairs of image units are calculated and blocked. After each color similarity value, we introduce the feature mapping method again in the following content, and 500 similarities are included in the 500-dimensional value mapping, and its feature is a binary space of 1. In the case of importance-based binary features (sbf), the feature dimension of each sample is 1000, i.e., 1000 pairs of points are selected from the preset position of the sample image. According to the feature mapping method described in this section, the importance mapping is mapped to a 1000-dimensional binary feature space containing 0.1. Finally, the two types of binary features are connected to form a 1500-dimensional binary feature vector. We verify the number of best fern classifiers for this fixed 1500-dimensional feature vector collected by each sample through experiments. The union of the six situations the authors have tried is as follows: 375 real time × 4 d/300 real time × 5 d/250 real time × 6 d/214 real time × 7 d/187 real time 166 real time × 8 d/9 d, of which 300 live × 5 d/250 live × 6 car group *d* has the detection effect, and the detection effect is similar, however, the final choice 250 is the real-time classifier. Each real-time classifier has 6-dimensional features divided into practice and testing, i.e., the total feature *n* is 1500 m = 250 sets, and each set features s = 6 dimensions. To better compare and understand the performance of the algorithms, this experiment still uses the det (detection error trade-off) curve described in the reference [Dal05] to evaluate the performance of the detector to compare the performance of the algorithms. The *x*-axis is the false positive window, and the *y*-axis is the error rate. Obviously low detection rate and low fppw are the manifestations of good detection results. The leakage rate and false alarm rate are calculated by the following formula:

(14) $$\begin{array}{c} miss\;rate=\frac{FalseNeg}{TruePos+FalseNeg}\text{,}\\ FPPW=\frac{FalsePos}{TrueNeg+FalsePos}\text{.} \end{array}$$

Figure 4 shows the algorithm RANCS-SBF + Ferns and algorithm HOG + SVM. In our experiments, we compared the proposed rancs-sbf function with the following four other function descriptors. In the case of local binary features, using the lbp feature descriptor in the literature, good detection results are obtained. The gradient histogram function is proposed by Dalal (hog). The rcs-lbp function of color and texture is proposed by Zhang et al., and the main function is proposed by Zott et al. The above four features have been fully detected in pedestrian detection, and the det curve corresponding to these four features is shown in the figure. For more specific detection test curves, one can refer to the literature corresponding to the above four characteristics. The Randafern classifier is used to select the classifier, and the support vector machine classifier is used for the other four algorithms. The final result is shown in the figure. It can be seen from the figure that, compared with the other four functions, the human detection algorithm of “rancs-sbf function + Randafern classifier” the authors proposed has obtained a lower detection rate and false alarm rate.

### 3.3. Visual Image Recognition Based on Particle Swarm Optimization

In the particle smoothing framework, the division and stability of the features of each visual integrated view of the particles are enhanced, and the fusion algorithm of visual feature weights and the realization of visual features are adjusted based on the optimization of particle groups. By changing the scene with the correct value, adapting to change is the realization of the goal. The characteristic of comprehensive observation is that other goals and backgrounds are the most distinctive. According to research and analysis, under the framework of particle filter theory, the multivision feature weight adaptive fusion tracking algorithm can be described as follows:

1. Initialization: use the *k* command to perform initial distribution according to frame 1 *px* state sample set initial 011, niixn initial. The initial visual feature synthesis weight of 1 m or more is 4.30.
2. Because of the transition model and particles, the transition of the particle state is usually very high, and the state is a random quantity. Taking this value, based on the optimization of the particle group in the latter part, the collection of particles is set as the target position as much as possible, and the minimum value is set as the local sample convergence of the particles.
3. The particle sample based on particle group optimization is a collection of particles in the largest area (for example, the largest area) to obtain a more effective coverage target particle sample strategy based on the particle group optimization strategy.
4. Calculate the smoothness of the particles in the visual feature frame and each observation probability of each particle.
5. Particle authority “ikw” calculation: depending on the result, the sensory feature is the most important value combination. According to the remaining visual features, the observation probability, the calculated particle authority, and naturalization are increased.
6. Target state and visual feature fusion output and calculate the best estimate of *k* instantaneous target state.
7. Respecimen: the re-extracted *n* particles form a set of new particles. With the concentration of new particles, each particle has the same number of permissions.

The proposed feature value based on particle swarm optimization is not so much an adaptive particle smoothing visual tailing algorithm; however, it is a part of the adaptive particle smoothing visual tailing algorithm. It is the first part of using the particle swarm optimization algorithm to improve the reference particle smoothness. Particle swarm optimization improves the effectiveness of the algorithm's particle samples. The second improvement area can follow the scene by changing the permissions of each visual feature and adjust the adaptability of the algorithm to implementation through particle swarm optimization. Below, the authors analyzed the following two aspects: the effectiveness of the particle sample enhancement algorithm through the particle swarm optimization analysis experiment is based on the effectiveness of the particle swarm optimization technique to achieve particle samples. Through our pursuit, we analyzed the improved algorithm of smoothing experiment based on the original discussion of standard particle smoothing. In the experiment, these three algorithms use the same parameter configuration. In other words, the number of particles is 100, and the weight of the two features is fixed to 0.5 according to the color feature of the gradient and the edge history feature.

Figure 5 shows the smooth trailing algorithm of particles based on Karlman's smooth prediction sample, and it also shows the tracking result of the tennis player's forehead. The number of frames in the figure shows the typical tracking result. In the figure, the tracking accuracy is greatly improved. Basically, all particles attract the target well around the target, and then, they distribute the experimental state. It is the ukf prediction of particle smoothing. Use the latest observational information and integrate it into the important suggestion distribution to enhance the effectiveness of smooth particle samples. The tracking process uses two tracking functions, namely the gradient-based gray histogram and edge histogram, to track pedestrians in the infrared scene. To verify the effectiveness of the proposed algorithm, we chose a scenario. However, it is obvious that when only the features of the gray histogram are applied, tracking drift will occur when two pedestrians meet. The three figures show that these three algorithms effectively follow and target pedestrians, and the figure that can be clearly understood is the constant trajectory of the figure below. The figure is a good tracking result, and because the algorithm embodied is the effectiveness of tailing, the trailing error depends on the three algorithms we summarized. As shown in the figure, the tracking algorithm we proposed has a smaller center tracking error.

Figure 6 shows the change curve, where in the multifeature weight adaptive tracking algorithm, the weights of the gradient-based edge direction histogram function, and the gray level histogram function are adaptively adjusted according to the movement of the target. From the first frame, we can see that the weight of the feature based on the gradient of the edge direction histogram is initialized to 0.72, and the weight of the gray feature is initialized to 0.28. It can be seen from the subsequent movement of the weight adjustment curve that the weight initialization strategy the authors proposed earlier is effective. In general, the overall particle optimization strategy the authors proposed allows the adaptive adjustment of visual feature weights throughout the tracking process.

## 4. Experimental Verification and Data Analysis of Athlete Detection

### 4.1. Experimental Scene Settings

In this paper, in the research based on the recognition method of the acceleration of the lower limbs to the pedestrian's heart, the pedestrian's behavior is analyzed from the side view, and the hypotheses proposed for the subject and the experimental scene are as follows:

1. Research object: this research's object is healthy, well-structured people without physical diseases, especially people with healthy lower limbs and normal walking function
2. Background photography: although there is no complicated background interference and the restrictions are not completely eliminated, the background of the laboratory is slight background interference and light changes
3. Shooting angle: in a horizontal angle, the camera lens keeps parallel to the travel path of the subject
4. Walk only when there is one target in the field of vision, and walk normally according to their daily walking habits

Pedestrians move in the walking direction at a normal walking speed. The camera remains still, and the lens remains parallel to the walking direction. Create an experimental website, collect walking video information, and process the collected video sequences according to the methods described.

### 4.2. Experimental Data Collection

First, briefly introduce the hardware and software used in the experiment. The image processing software mainly divides the walking targets according to the order of the video and realizes the positioning of the relevant points of the lower limbs of the human body. The processing software for this image processing in this experiment is matlab7.10.0. We introduce mathematical software and algorithm compilation to make the data more real for image processing and data analysis. Computer: the computer used in the experiment is a 32-bit computer equipped with Win7. Video shooting tool: the video shooting tool used in the experiment is a Canon110, which is camera with 4 × optical zoom and 4 × digital zoom. The focal length was preset during the shooting, and digital zoom and optical zoom did not occur during shooting. According to the preface, Kosuke is one of the relevant parameters to solve the heart acceleration of the lower limbs in walking. In practical applications, only the image, video, and anatomical structure of the human body are obtained from the acquisition of leg length parameters. It is understood that even for normal people participating in the experiment, there is a proportional relationship between the leg length and the fixed height of the human body. The length of the thigh is hl 25.01, and the length of the thigh is hl 246.02. The order is an image, and the source of the height of the human body is an important experiment content. The method of restoring height is introduced; however, the figure is an optical circuit diagram of restoring height, which lists the statistical results of the experiment. In actual experiments, if the reference object in the plane composed of the center of the human body and the direction of travel is selected and the actual height is known in advance, the statistical result of the height reduction of the target height table of the human body can be estimated. The statistics of height reduction are shown in Table 1.

By collecting the sequence of walking images, processing and adjusting the minute frames, a possible background model of the contour image sequence can be constructed, and to extract the period and key frames, the binary image on the human body can be used. By obtaining the effective expected area deducted and divided in the operating background, the relevant points of the lower body of the human body in the effective expected part are obtained to confirm the information of the lower limb joints of the human body that is walking normally. By walking to the image of the human body, we found the relative point positioning of the lower limb posture in sequence and matched the tendency of swinging to the lower body of different human bodies. In the initial stage of support selection, the rhythm of the movement is matched at the middle and end of the support, and the symmetry of the person's walking movement (the way of supporting rotation and supporting leg is different), the left leg is shown in the figure. The human body swells under the support of the right leg and the swing of the right leg, showing the general law of the working posture of the lower limbs in these three postures. The joint angles of these three postures are all 10 people.

Table 2 shows the statistics of the joint angle of the thigh during the pedestrian support phase.

The statistical joint angle information in the above table provides a basis for solving dynamic parameters (such as lower limb angular velocity and angular acceleration). According to the analysis of human walking characteristics in the original content, the change of joint angle is the result of angular velocity, and the change of angular velocity will also cause angular acceleration. The statistical table of angles of calf joints in different pedestrian support phases is shown in Table 3.

### 4.3. Comparative Verification and Result Analysis

The three pedestrians, a, *b*, and *c*, who entered the experimental site were measured multiple times, and the data obtained each time were summarized. During the measurement, the laboratory workbench did not move. The relevant motion parameters of each subject were statistical data. These motion parameters include the angular velocity, angular acceleration, and center petal acceleration of the thigh and calf. The statistical results are displayed on the table. Each parameter of the pedestrian is shown in Table 4. Pedestrian B parameters are shown in Table 5.

We compare and analyze the data collected in the statistical table with the information in the statistical database. In actual situations, pedestrians are a, *b*, and *c*, respectively. By comparing the experimental measurement results with the data collected from the information database before the verification experiment, the four-line data of passer-by *a* can be found by the sequence of further approaching the database and the remaining four-line data. The purpose of originator *a* can only be identified as the closest to the data corresponding to level 3. The data in the database of pedestrian *b* and pedestrian *c* is relatively close to the data verified in the experiment, and it can be identified. If the measurement is not accurate, then it may interfere with recognition. However, in general, the data shown in the table is a rough idea. Pedestrian *C* parameters are shown in Table 6.

For each motion parameter of pedestrian *a* in the table, firstly, consider the data string of height *h*. Only sequence 3 and sequence 5 are the closest in the table. According to the statistical calculation of data errors, the experimental result is greater than the positive value of the daily basic data. Otherwise, it is negative. In sequence 3, the errors of the five experimental data of pedestrian *a* are +0.0002, −0.0006, −0.0003, +0.0028, and +0.0001. For sequence 5, they are −0.0005, −0.0013, −0.0010, +0.0021, and −0.0006. In the experimental statistical database, the tables of level 3 acceleration and level 5 acceleration are the calculation data of angular acceleration and cardiac acceleration, respectively. The result of sequence recognition is the error size of the data, and the total difference between order 3 and order 5 is the most reasonable. After comparison, it is found that the third-order data is the most reasonable. But in reality, according to the model data of A in the next three stages, pedestrian data can achieve the purpose of recognition. Since the statistics of pedestrian *b* and pedestrian *c* are very close, the error is not clear, and if misidentification occurs during the experiment, it is difficult to identify. However, if the individual differences are relatively clear, they will be identified.

## 5. Conclusion

However, with the development of science and technology and the improvement of computerization, people can walk according to the demand for information security, especially in public sensitive areas, and according to the demand for foot pressure measurement analysis and recognition technology. The research method has been continuing for a long time. The measurement-based foot pressure recognition technology has good accuracy, high decoding rate, and high reliability, however, it cannot be applied to high transmission, except for equipment. In this article, we propose a walking state recognition method, which is characterized by acceleration from the lower limbs to the heart. To realize the above method, firstly, it is necessary to analyze the movement law of the lower limbs of the human body and establish a dynamic model of the lower limbs of the human body. Propose a method based on the acceleration of the lower limbs to the heart to recognize the walking state. The effectiveness is analyzed. Next, the authors analyzed the advantages and disadvantages of many background modeling methods to obtain a more accurate background model. We propose a background modeling method that combines Gaussian mixture model and frame difference method. Next, on the basis of the obtained background model, the division and characteristics of the target traveling along the human body image are extracted, and the lower body of the human body will be equivalently applied to the gyration motion and the Milky Way viewpoint. Among them, on the basis of combining the symmetry of the periodic walking motion, the position of the correlation point of the lower limb lifted up on one side for walking is found. Finally, the experimental platform is constructed and the motion parameters of the lower limbs are constructed. Collect and calculate the central acceleration of the lower limbs. By collecting the motion parameter data of multiple experimental groups, the authors clarified the differences between individuals and proved that the central acceleration of the lower limbs can be used as an auxiliary identification feature in the identification method.

## Figures and Tables

**Figure 1:** Training a single fern classifier.

**Figure 2:** Multiclass single classifier.

**Figure 3:** Binary feature extraction based on saliency map. (a) Original image. (b) Saliency image.

**Figure 4:** Algorithm RANCS-SBF + Ferns and algorithm HOG + SVM.

**Figure 5:** Insensitive particle filter.

**Figure 6:** Center tracking error of PF-PSO-FW, SPSO, and PF-PSO-AW.

**Table 1:** Statistics of height reduction.

Sequence	Actual body (cm)	Restore height (cm)
1	1.822	1.8318
2	1.720	1.7191
3	1.653	1.6505
4	1.781	1.7819
*5*	1.644	1.6512
6	1.815	1.8226
7	1.783	1.7914
*S*	1.625	1.6336
9	1.754	1.7622
10	1.793	1.8053

**Table 2:** Statistics of thigh joint angles in different pedestrian support stages (°).

Sequence	Early support	Support midterm	End of support
1	−6 20	25.66	25.31
2	−6.95	20.85	20.73
3	−2.64	21.46	21.18
4	−5.23	23.44	23.26
5	−3.86	22.51	22.33
6	−6.08	24.02	23.84
7	−5.92	24.89	24.72
8	−5.88	22.67	22.43
9	−2.78	22.12	21.88
10	−4.96	24.37	24.06

**Table 3:** Statistical table of angles of calf joints in different pedestrian support phases (°).

Sequence	Early support	Support midterm	End of support
1	−43.60	−66.88	−0.28
2	−40.90	−55.24	−1.43
3	−46.05	−63.22	−1.02
4	−42.85	−60.52	−1.03
5	−44.56	−65.07	−1.26
6	−43.27	−64.75	−1.38
7	−45.34	−62.66	−0.57
8	−41.76	−59.69	−0.92
9	−41.23	−56.62	−1.37
10	−45.82	−63.77	−1.18

**Table 4:** Each parameter of pedestrian.

H(m)	Φ_1_(rad/s^2^)	*φ*_1_^″^(rad/s^2^)	*a*_1_(m/s^2^)	Φ_2_(rad/s^2^)	*φ*_2_^″^(rad/s^2^)	*a*_2_(m/s^2^)
1.6507	1.299	−14.725	3.462	1.508	27.351	5.883
1.6499	1.301	−14.731	3.480	1.516	27.357	5.876
1.6502	1.287	−14.693	3.470	1.536	27.402	5.901
1.6533	1.172	−12.066	2.798	1.467	28.063	5.972
1.6506	1.301	−14.719	3.485	1.513	27.358	5.882

**Table 5:** Pedestrian B parameters.

*H* (m)	Φ_1_(rad/s^2^)	*φ*_1_^″^(rad/s^2^)	*a*_1_(m/s^2^)	Φ_2_(rad/s^2^)	*φ*_2_^″^(rad/s^2^)	*a*_2_(m/s^2^)
1.7910	1.325	−12.258	3.254	1.497	27.358	6.279
1.7935	1.341	−12.272	3.290	1.503	27.372	6.308
1.7918	1.322	−12.078	3.196	1.498	27.420	6.332
1.7962	1.297	−11.984	3.104	1.495	27.638	6.381
1.7913	1.301	−12.085	3.137	1.502	27.536	6.376

**Table 6:** Pedestrian *C* parameters.

H(m)	Φ_1_(rad/s^2^)	*φ*_1_^″^(rad/s^2^)	*a*_1_(m/s^2^)	Φ_2_(rad/s^2^)	*φ*_2_^″^(rad/s^2^)	*a*_2_(m/s^2^)
1.7998	1.297	−12.039	3.123	1.493	27.556	6.377
1.8012	1.282	−11.997	3.112	1.499	27.637	6.401
1.7952	1.325	−12.002	3.238	1.505	27.340	6.309
1.8078	1.267	−11.863	3.082	1.489	27.742	6.405
1.7983	1.316	−11.952	3.104	1.495	27.687	6.396

## Data Availability

The data used to support the findings of this study are available from the author upon request.
